The article "Effect of Mirena Intrauterine Device on Endometrial Thickness, Quality of Life Score, and Curative Effect in Patients with Perimenopausal Abnormal Uterine Bleeding" was published in 2022. Journal: Comput Math Methods Med.

# Effect of Mirena Intrauterine Device on Endometrial Thickness, Quality of Life Score, and Curative Effect in Patients with Perimenopausal Abnormal Uterine Bleeding

**DOI:** 10.1155/2022/5648918

**Published:** 2022-09-30

**Authors:** Ying Yu, Zhi Zhou, Liping Wang, Jie Liu

**Affiliations:** ^1^Reproductive Medicine Center, Huanggang Central Hospital of Yangtze University, Huanggang, Hubei 438000, China; ^2^Obstetrics and Gynecology Department, Tuanfeng Maternal and Child Health Hospital, Huanggang, Hubei 438000, China; ^3^Obstetrics and Gynecology Department, Huanggang Central Hospital of Yangtze University, Huanggang, Hubei 438000, China

## Abstract

**Objective:**

To study the effect of Mirena intrauterine device (IUD) on endometrial thickness, life quality score, and curative effect in patients with perimenopausal abnormal uterine bleeding.

**Methods:**

Eighty patients with perimenopausal abnormal uterine bleeding cured from January 2020 to December 2021 were enrolled as the object of study. According to random number table, the patients were classified into the study (*n* = 40) and control (*n* = 40) groups. The control cases were cured with medroxyprogesterone. The study cases were cured with Mirena IUD. The effective rate of clinical therapies was evaluated after 3 months of treatment. The endometrial thickness, menstrual volume score, and life quality score (WHOQOL-BREF) was measured after 1 month, 2 months, and 3 months of treatment.

**Results:**

The effective rate of patients with Mirena IUD for 3 months was higher compared to the control group (*P* < 0.05). The endometrial thickness and menstrual volume scores of study cohort after 1 month, 2 months, and 3 months following treatment were remarkably lower than those before treatment (*P* < 0.05) and were considerably lower than those of control cohort (*P* < 0.05). The hemoglobin level of the studied cases after 1 month, 2 months, and 3 months after therapy was remarkably upregulated (*P* < 0.05) and was greatly higher compared to the controlled cases (*P* < 0.05). After 3-month treatment, the WHOQOL-BREF score of the study group was higher compared to the control group (*P* < 0.05).

**Conclusion:**

The Mirena IUD is far more effective in the treatment of perimenopausal abnormal uterine bleeding and is helpful in reducing the thickness of the endometrium. Patients' menstrual flow can be controlled, and anemia can be corrected; thus, patients improve their quality of life and health status and can be considered for further promotion.

## 1. Introduction

Perimenopausal period is the temporary period from the decline of female ovarian function to 1 year after menopause [1]. The ovarian function of perimenopausal women gradually declined, the sensitivity and response of ovaries to pituitary gonadotropin decreased, and the negative feedback of estrogen and progesterone caused the increase of gonadotropin level [2]. The levels of thyroid-stimulating hormone (TSH) and luteinizing hormone (LH) increased remarkably, and the reflex of estrogen in the body increased, but it could not form a preovulatory peak, follicular development and maturation reduced the disturbance of ovulation, and the level of progesterone was low [3]. The endometrium is affected by a single estrogen showing obvious proliferative changes, and the endometrium cannot be well transformed into the secretory phase [4–6].

The definition of abnormal uterine bleeding is inconsistent with any of the four items of normal menstrual frequency, regularity, menstrual duration, and menstrual bleeding volume, which comes from abnormal bleeding in the uterine cavity [7]. Under normal circumstances, the menstrual cycle of women is under the action of neuroendocrine regulation mechanism of reproductive axis (also called hypothalamus-pituitary-ovary axis), and endometrium changes periodically and falls off. Under normal circumstances, the menstrual cycle appears regularly, which the average time is 23-37 days with menstrual volume of 20~60 ml for menstrual period of 3-7 days [8]. The hypothalamic-pituitary-ovarian system in perimenopausal women is prone to disruption due to reduced ovarian sensitivity and response to gonadotropins. The ovarian function shows the trend of decline, which follicular growth and development is relatively slow and ovulation dysfunction occurs, resulting in a significant decrease in progesterone secretion [9]. Endometrium is only affected by estrogen, and the lack of progesterone antagonistic effect and estrogen breakthrough uterine bleeding occurs, which is more likely to cause perimenopausal abnormal uterine bleeding [10–12]. The main clinical manifestations are irregular menstrual cycle, remarkably increased menstruation, prolonged menstruation, endless dripping, and secondary anemia accompanied by systemic symptoms such as dry skin, hot flashes, chest tightness, and irritability [13].

The therapeutic guidelines for perimenopausal abnormal uterine bleeding are to stop bleeding and correct anemia, to regulate the menstrual cycle, to prevent endometrial cancer, and to promote quality of life [14]. The traditional nonoperative treatment is mainly oral hormone drugs, such as medroxyprogesterone [15]. Medroxyprogesterone is a progesterone derivative of 17-a hydroxyprogesterone, which is a synthetic luteal progesterone. In the treatment of perimenopausal abnormal uterine bleeding, high levels of medroxyprogesterone cause endometrial atrophy and inhibit the formation of local blood vessels in the endometrium, thereby altering the uterine microenvironment and promoting blood clotting [16]. Mirena, also known as levonorgestrel intrauterine birth control system (LNG-IUS), is an efficient and safe T-shaped plastic stent contraceptive device produced by Bayer Pharmaceutical Company of Germany. It was allowed to be adopted in 1995 and has been widely applied in many European countries since 2009. Mirena contains 52 mg levonorgestrel. Its unique design structure enables it to release levonorgestrel at a uniform rate at the dose of 20*μ*g/24 h, which can be maintained for about 5 years. The levonorgestrel drug and the contraceptive ring are capable of acting directly on the uterine cavity, causing the expression of progesterone and estrogen receptors to be downregulated. The endometrium becomes less sensitive to estrogen and progesterone and therefore gradually shrinks and thins, eventually leading to reduced menstruation. It can be adopted for contraception and treatment of menorrhagia caused by nonorganic diseases [17]. Only 10% of levonorgestrel is absorbed into the blood circulation, so Mirena has almost no endocrine effect on ovarian function, and patients with perimenopausal abnormal uterine bleeding do not need long-term oral hormone drugs [18]. Under this background, it is very necessary to carry out related research, which can clarify the role of Mirena intrauterine device (IUD) when treating perimenopausal patients with abnormal uterine bleeding, which will provide a certain basis for clinicians to judge the condition of patients. Based on this, this study focused on 80 cases of perimenopausal abnormal uterine bleeding cured in our hospital from January 2020 to December 2021.

## 2. Patients and Methods

### 2.1. General Information

Eighty patients with perimenopausal abnormal uterine bleeding cured from January 2020 to December 2021 were enrolled in our hospital as the object of study. Eighty patients were arbitrarily classified into the study (*n* = 40) and control (*n* = 40) groups. The age of study cases was 41-55 years old; their average age was 45.36 ± 4.22 years old, and the average course of disease was 7.15 ± 4.38 months. The age of control cases was 40-56 years old; their average age was 45.42 ± 4.17 years old, and the average course of disease was 7.19 ± 4.41 months. There exhibited no significant difference in sex, age, and course of disease (*P* > 0.05). This study was approved by the Medical Ethics Society of our hospital. All patients have signed an informed consent form. Inclusion criteria are as follows: (1) the cases who met the diagnostic criteria of perimenopausal period, and their age was in perimenopausal period. Premenstrual syndrome (PMS) symptoms during perimenopause can mirror those of menopause symptoms, confusing women as to what exactly are they suffering from and what initiatives they should take to find relief. It usually starts in your mid-40s, but it can start earlier. Completing menopause before age 40 is called premature menopause; (2) the patients who were diagnosed by hysteroscopy or directly diagnosed as perimenopausal abnormal uterine bleeding after uterine curettage; (3) the patients who had no heart, liver, kidney, and other medical complications; (4) the patients without fertility requirements; (5) the patients who could successfully complete follow-up; (6) the patients cured with Mirena and medroxyprogesterone.

Exclusion criteria are as follows: (1) pregnancy-related bleeding; (2) reproductive organ tumor; (3) systemic inflammatory reaction; (4) coagulation dysfunction and liver, kidney, endocrine diseases, and abnormal development of reproductive organs; (5) irregular vaginal bleeding caused by exogenous hormones and foreign bodies; (6) gynecological infection; (7) urinary system infection; (8) history of infectious abortion within 3 months; (9) hypersensitivity to levonorgestrel and medroxyprogesterone.

### 2.2. Treatment Methods

#### 2.2.1. Technical Route

The technical route of this research is displayed as indicated in Figure 1. Patients were recruited into the groups. The control group was given implementation of medroxyprogesterone treatment. The research group was given implementation of the treatment of Mirena IUD. The effective rate of clinical treatment after 3-month treatment and the endometrial thickness, menstrual volume score, and quality of life score (WHOQOL-BREF) were compared at 1 month, 2 months, and 3 months after treatment.

#### 2.2.2. Intervention Program

After the patient completed blood routine, urine routine, blood coagulation function, liver and kidney function examination, and B-ultrasound to determine the thickness of endometrium, routine diagnostic curettage was performed. Additionally, the scraped endometrial tissue was fixed with 10% formaldehyde solution and sent for pathological examination. Endometrial malignant and precancerous lesions were excluded according to the results of pathological examination.

1. Control group: medroxyprogesterone (Zhejiang Xianwei Pharmaceutical Co., Ltd., specification: 2 mg/tablets) treatment; oral medroxyprogesterone 8 mg (four tablets a day) half a month after endometrial tissue curettage. The cases stopped taking medicine for 10 days and waited for endometrial exfoliation and bleeding. From the first day of bleeding, the cases would wait for half a month to start taking medicine. The continuous treatment should be last for 3 months
2. Study group scheme: Implement Mirena LNG-IUS was produced by Bayer, Germany, with specification 52 mg/branch. Its main composition is the chemical name of levonorgestrel D (–)–17*α*–-ethynyl-17 *β*-hydroxy-18-methylestrost-4- alkene-3- ketone; and the molecular formula is C_21_H_28_O_2_. The core of Mirena is a white or quasi-white cylindrical structure, and the outer cover is fixed to the T-shaped longitudinal arm with an opaque film. The horizontal arm is folded away and placed in the placer. After the gynecological examination, the size and position of the uterus were determined. Mirena ring was placed in the uterus on the fifth day after curettage. After placing Mirena, the patients stayed in bed for 2 hours to observe the adverse reactions such as fever, abdominal pain, or vaginal bleeding. Regular follow-up observation was conducted after placement; if there was no obvious discomfort in the treatment effect of the patient and the conscious effect was satisfactory, it can be taken out when the hormone level of the patient has reached menopause. Regular follow-up visits include understanding the patient's condition and assessing treatment; understanding the patient's behavioral changes and adjusting nonpharmacological treatment plans; understanding the patient's visits and medication use and evaluating the effectiveness of medication; supervising the patient's regular blood pressure, blood glucose, lipid, and related complications checks; and understanding and checking the patient's self-management. It can be removed at any time when the patient feels obviously uncomfortable or the therapeutic effect is not obvious during treatment

### 2.3. Observation Indicators

1. The effective rate of clinical treatment after 3 months of treatment was studied: from the beginning of the treatment, the patients will be followed up every month, and the patients will be informed to come to the hospital for reexamination on time. The curative effect was observed and blood routine examination and B-ultrasound were performed. The hemoglobin level and the thinning of endometrium were observed. In the meantime, the patient was asked whether there was irregular bleeding, nausea, vomiting and other discomfort, anemia, and if symptoms of anemia and fatigue were improved. The criterion for efficacy is return to normal menstrual cycles lasting 3-5 days each cycle after treatment. The patients with significantly reduced or amenorrhoeic menses were deemed to be effective. Conversely, the patients whose vaginal bleeding did not change or worsened after treatment were considered ineffective
2. The thickness of endometrium before treatment, 1 month, 2 months, and 3 months after treatment was detected by color ultrasound
3. The menstrual volume scores before treatment, 1 month, 2 months, and 3 months after treatment were compared. Menstrual bleeding chart (PBLAC) was adopted to evaluate in this investigation [19]. PBLAC score (1) 0: no menstruation (amenorrhea), (2) 1~10: drip bleeding, (3) 11~30: decreased menstruation, (4) 31~100: normal menstruation, (5) 100~150: menorrhagia, and (6) >150: menorrhagia
4. The hemoglobin level before treatment, 1 month, 2 months, and 3 months after treatment: venous blood was drawn to detect blood routine and count the amount of hemoglobin
5. The life quality score: WHOQOL-BREF score was adopted to evaluate the quality of life. The WHOQOL-BREF scale included 26 items, including physiology, psychology, social relations, and environment [20]. Each entry would be scored 1-5 points from light to heavy, and 3 items needed reverse score. The score of each field = the average score of the field to which it belongs is ^∗^ 4. The higher the score in the field, the better the quality of life in the corresponding field

### 2.4. Statistical Analysis

The statistical analysis was calculated using SPSS24.0 software, and the statistical graphics were drawn by GraphPad Prism8.0. The measured data in accordance with normal distribution were presented by mean ± standard deviation ($\bar{x}\pm \text{s}$). Paired sample *t*-test was adopted for intragroup comparison, and independent sample *t*-test was applied for intergroup comparison. *P* < 0.05 exhibited statistically significant. If it was not consistent, it was presented by the median (lower quartile to upper quartile). Paired sample nonparametric test was adopted for intragroup comparison, and independent sample nonparametric test was used for intergroup comparison. The grade data were tested by FISHER accurate method. *P* < 0.05 exhibited statistical significance.

## 3. Results

### 3.1. Effective Rate of Clinical Treatment after 3 Months of Treatment

After 3 months of treatment, the clinical effective rate of the study group was higher compared to the control group (*P* < 0.05, Table 1). The data indicated that Mirena IUD had more effective than medroxyprogesterone.

### 3.2. The Thickness of Endometrium before Treatment and 1 Month, 2 Months, and 3 Months after Treatment

Before treatment, there exhibited no significant difference in endometrial thickness (*P* > 0.05). The thickness of endometrium in the study group after 1 month, 2 months, and 3 months treatment were remarkably thinner than that before treatment (*P* < 0.05), and they were greatly thinner lower than those in the control group (*P* < 0.05), as indicated in Table 2. The current results suggested that Mirena IUD could inhibit the growth of the thickness of endometrium compared with medroxyprogesterone treatment.

### 3.3. The Menstrual Volume Scores before Treatment and 1 Month, 2 Months, and 3 Months after Treatment

Before treatment, there exhibited no significant difference in menstrual volume score (*P* > 0.05). The menstrual volume scores of the study group at 1 month, 2 months, and 3 months after treatment were remarkably lower than those before treatment (*P* < 0.05), and they were remarkably lower than those in the control group (*P* < 0.05), as indicated in Table 3. The current results suggested that Mirena IUD could reduce the menstrual volume compared with medroxyprogesterone treatment.

### 3.4. The Hemoglobin Level before Treatment and 1 Month, 2 Months, and 3 Months after Treatment

Before treatment, there exhibited no significant difference in hemoglobin content (*P* > 0.05). The hemoglobin level of the study group after 1 month, 2 months, and 3 months of treatment was remarkably higher than that before treatment (*P* < 0.05), and they were remarkably higher than those in the control group (*P* < 0.05, Table 4). The current results showed that Mirena IUD could reduce the menstrual volume in order to maintain higher hemoglobin level compared with medroxyprogesterone treatment.

### 3.5. WHOQOL-BREF Score

There exhibited no significant difference in WHOQOL-BREF score before treatment (*P* > 0.05). After 3 months of treatment, the WHOQOL-BREF score of the study group was higher compared to the control group (*P* < 0.05, Table 5). The current results showed that Mirena IUD could improve the life quality of patients.

## 4. Discussion

Since the implementation of family planning in China, the aging population has also increased accordingly, and the number of people entering menopause is becoming larger and larger. According to a survey from the United Nations, the number of perimenopausal people was expected to reach 197 million by 2020 [21]. There is no clear age limit for perimenopausal period, and the time of ovarian function decline in women is different. Perimenopause means “around menopause” and refers to the time during which your body makes the natural transition to menopause, marking the end of the reproductive years [22]. Before menopause, some patients will develop symptoms associated with ovarian decline. The main manifestations are mental and emotional irritability and sleep disorders [23]. Additionally, some patients will show sparse menstruation or dripping, which symptoms will make people more irritable and nervous. In the perimenopausal period, there will be some other physical discomfort, such as slow intestinal peristalsis, loss of appetite, and fatigue without any inducement. The decline in estrogen levels will increase the incidence of cardiovascular disease, and these subsequent symptoms and physical discomfort seriously plague perimenopausal women [24–28].

In the perimenopausal period, the follicles in the ovary are gradually exhausted, and the follicles are an important source of estrogen secretion in the female body [29]. Perimenopausal endometrium is stimulated by single estrogen for a long time. However, the proliferative endometrium cannot be converted to secretory phase due to the decrease of progesterone level, and the blood vessels and stroma of endometrium are easy to break and bleed [30]. Therefore, women approaching menopause are particularly prone to irregular uterine bleeding. Abnormal uterine bleeding is one of the most common gynecological problems in perimenopausal women. Most of the women approaching menopause are caused by abnormal uterine bleeding caused by ovulation disorders [31]. In the United States, gynecological diseases, including abnormal uterine bleeding, are the leading cause of hospitalization for women aged 45-54, accounting for 14% of the total hospitalization rate [32]. The annual cost of treatment for abnormal uterine bleeding is about $100 million [33]. Therefore, our country will spend more and more on treating the diseases of perimenopausal women with the increase in the number of postmenopausal people. How to manage abnormal uterine bleeding effectively and economically is an important problem what we are facing.

Clinical studies have indicated that medroxyprogesterone could be adopted to treat perimenopausal abnormal uterine bleeding, but patients had varying degrees of treatment dependence, easy to relapse after treatment [34]. Moreover, it is not easy for patients to master the method of medication, and it is difficult to use drugs regularly. Long-term unregulated use of medication is not conducive to improving the disease and can lead to recurrence or even aggravation. In addition, previous studies have indicated that long-term oral hormone drugs can increase the incidence of cardiovascular and cerebrovascular diseases, endometrial cancer, and breast cancer to a certain extent, which will bring great physical pain and psychological problems to patients to a certain extent [35]. Mirena LNG-IUS is produced by Bayer and contains 52 mg levonorgestrel, which can stably and slowly release levonorgestrel [36]. Through a sustained release system, levonorgestrel is continuously released into the target organ, where it is absorbed through the basal capillary network of the endometrium, inhibiting the synthesis of endometrial estrogen receptors, and thus antagonizing endometrial hyperplasia [37]. Therefore, a single-center randomized controlled trial was conducted to explore the effects of Mirena IUD on endometrial thickness, quality of life score, and efficacy in patients with perimenopausal abnormal uterine bleeding.

Our results displayed that the effective rate of patients with Mirena IUD for 3 months was greatly higher compared to the control cohort. The endometrial thickness and menstrual volume scores of study cohort after 1 month, 2 months, and 3 months following treatment were remarkably thinner than those before treatment and were considerably thinner than those of control cohort. The hemoglobin level of the studied cases after 1 month, 2 months, and 3 months after therapy was remarkably upregulated (*P* < 0.05) and was greatly higher compared to the controlled cases. After 3-month treatment, the WHOQOL-BREF score of the study group was higher compared to the control group. The results of this study further confirmed that Mirena IUD was effective when treating perimenopausal patients with abnormal uterine bleeding, which was more beneficial to enhance the thickness of endometrium, control menstrual volume, correct anemia, and promote the quality of life. This is mainly because Mirena is a new type of contraceptive, which combines ordinary birth control device with oral contraceptive, giving full play to their advantages [38]. The females with abnormal uterine bleeding in perimenopausal period are older and have relatively poor tolerance to drug metabolism and side effects. The long-term use of hormone drugs will lead to cardiovascular disease, osteoporosis, insomnia, depression, and other adverse events [39]. Moreover, 20ug levonorgestrel is released daily and directly acted on the uterine cavity following placement in the uterine cavity. Because the concentration in the serum is very low, it has almost no effect on the ovaries, and the systemic side effects will be greatly reduced.

Zhao et al. conducted a questionnaire survey on 1021 Chinese women who used Mirena in 12 different cities [40]. That results suggested 41% of the patients adopted the Mirena Ring because of abnormal uterine bleeding, most of the patients had less uterine bleeding during the use, and more than 90% of the patients consciously had better outcomes. A study on the treatment of bleeding with medroxyprogesterone and medroxyprogesterone indicated that the Mirena group remarkably improved the hyperplasia of endometrium than the medroxyprogesterone group and the cure rate was higher than the progesterone treatment. Several studies have indicated that the endometrial thickness of the Mirena group will be further thinned during subsequent follow-up. In addition, the satisfaction of the patients and the efficacy of treatment were remarkably enhanced compared with the medroxyprogesterone group [41]. This has been consistent with the results of this study. Therefore, it can be considered that Mirena has the advantages of convenience, high compliance, and less systemic side effects when treating perimenopausal abnormal uterine bleeding. The shortcomings of this study are the small number of observed factors and the small sample size, and further clinical studies with large samples are needed.

In summary, the Mirena IUD is far more effective in the treatment of perimenopausal abnormal uterine bleeding and is helpful in reducing the thickness of the endometrium. Patients' menstrual flow can be controlled, and anemia can be corrected, and thus patients improve their quality of life and health status and can be considered for further promotion.

## Figures and Tables

**Figure 1:** Technology roadmap.

**Table 1:** The effective rate of clinical therapies after 3 months of treatment.

Group	Effective (example/%)	Valid (example/%)	Invalid (example/%)	Effective rate of clinical treatment (case/%)
C group (*n* = 40)	24/60.00	7/17.50	9/22.50	31/77.50
R group (*n* = 40)	30/75.00	8/20.00	2/5.00	38/95.00
*χ* ^2^ value				0.119
*P* value				0.731

**Table 2:** The thickness of endometrium before treatment and 1 month, 2 months, and 3 months after treatment.

Thickness of endometrium (mm)	Before treatment	Treatment for 1 month	Treatment for 2 months	Treatment for 3 months
C group (*n* = 40)	13.54 ± 4.19	11.82 ± 3.11^∗^	8.99 ± 308	7.39 ± 2.25^∗^
R group (*n* = 40)	13.35 ± 4.12	9.69 ± 2.23^∗^	7.24 ± 2.02^∗^	5.11 ± 1.06^∗^
*t* value	0.204	3.520	3.004	5.798
*P* value	0.838	<0.01	0.004	<0.01

Note: ^∗^ was indicated that the values of after 1 month, 2 months, and 3 months of treatment were compared with that before treatment, *P* < 0.05.

**Table 3:** The menstrual volume scores before treatment, 1 month, 2 months, and 3 months after treatment.

Menstrual volume score (points)	Before treatment	Treatment for 1 month	Treatment for 2 months	Treatment for 3 months
C group (*n* = 40)	181.54 ± 15.19	115.82 ± 13.11^∗^	94.12 ± 8.39^∗^	78.19 ± 9.25^∗^
R group (*n* = 40)	181.38 ± 15.12	70.69 ± 11.03^∗^	65.14 ± 5.44^∗^	56.23 ± 8.35^∗^
*t* value	0.047	16.659	18.329	11.145
*P* value	0.963	<0.01	<0.01	<0.01

Note: ^∗^ was indicated that the values of after 1 month, 2 months, and 3 months of treatment were compared with that before treatment, *P* < 0.05.

**Table 4:** The hemoglobin level before treatment, 1 month, 2 months, and 3 months after treatment.

Hemoglobin content value (score)	Before treatment	Treatment for 1 month	Treatment for 2 months	Treatment for 3 months
C group (*n* = 40)	73.52 ± 9.12	80.24 ± 9.22^∗^	90.29 ± 9.64^∗^	97.59 ± 9.32^∗^
R group (*n* = 40)	73.49 ± 9.09	85.08 ± 10.13^∗^	99.31 ± 10.65^∗^	111.36 ± 10.14^∗^
*t* value	0.015	2.235	3.971	6.323
*P* value	0.988	0.028	<0.01	<0.01

Note: ^∗^ was indicated that the values of after 1 month, 2 months, and 3 months of treatment were compared with that before treatment, *P* < 0.05.

**Table 5:** The WHOQOL-BREF score before and after treatment.

WHOQOL-BREF score (score)	Before treatment	Treatment for 3 months	*t*	*P* value
C group (*n* = 40)	69.23 ± 8.37	82.09 ± 10.47	6.068	<0.01
R group (*n* = 40)	69.18 ± 8.42	102.25 ± 11.01	15.089	<0.01
*t*	0.027	8.392		
*P* value	0.979	<0.01		

## Data Availability

The datasets used and analyzed during the current study are available from the corresponding author upon reasonable request.
